# Progesterone Reduces ATP-Induced Pyroptosis of SH-SY5Y Cells

This article has been retracted.

**DOI:** 10.1155/2022/4827444

**Published:** 2022-08-12

**Authors:** Chang Cui, Xiaona Wang, Siyu Zhang, Hui Wu, Meijie Li, Luoxiao Dong, Chongshuai Yan, Dongliang Li

**Affiliations:** ^1^Department of Pathophysiology, School of Basic Medicine, Sanquan College of Xinxiang Medical University, Xinxiang, 453003 Henan, China; ^2^Pingdingshan Industrial Vocational and Technical College, Pingdingshan, 467000 Henan, China

## Abstract

**Aim:**

To investigate the mechanism of progesterone inhibiting the scorch death of SH-SY5Y cells induced by exogenous adenosine triphosphate (ATP).

**Methods:**

SH-SY5Y cells with good logarithmic growth were used in the experiment. The cells were randomly divided into 5 groups: normal control group, DMSO group, BBG group, ATP group, and ATP+progesterone group. The cell survival rate of each group was measured by CCK-8 method. The expressions of P2X_7_ receptor, caspase-1, caspase-11, and IL-1*β* were detected by western blotting.

**Results:**

(1) After SH-SY5Y cells were treated with ATP at different concentrations (1, 3, 6, and 9 mmol/L) for 2 hours, the cell survival rate decreased in a concentration-dependent manner compared with the normal blank group. The results showed that the optimal lethal concentration of ATP was 6 mmol/L. SH-SY5Y cells were preincubated with progesterone at different concentrations (3, 10, 30, and 100 nmol/L) for 30 minutes and then incubated with 6 mmol/L ATP. The cell survival rate of this group was significantly improved (*P* < 0.01). The optimal concentration of progesterone to improve cell survival and inhibit cell death was 30 nmol/L. (2) Compared to the control group, there was no significant difference (*P* > 0.05) in P2X_7_ receptor, caspase-1, caspase-11, and IL-1*β* with the DMSO group (0.001% DMSO, 24 h) and BBG group (bbg1 mmol/L, 24 h). (3) In the ATP group, the expression of P2X_7_ receptor and caspase-1 (the key protein of classical cell death pathway) increased significantly (*P* < 0.01), which was related to inflammatory factor IL-1*β* with consistent performance (*P* < 0.01). There was no significant change in caspase-11 (the key protein of nonclassical focal death pathway) (*P* > 0.05). (4) The expression of P2X_7_ receptor, caspase-1, and inflammatory factor IL-1*β* in the progesterone+ATP group was significantly downregulated (*P* < 0.01). There was no significant change in caspase-11 (*P* > 0.05).

**Conclusion:**

Certain dose of progesterone can inhibit the focal death of SH-SY5Y cells induced by extracellular high concentration ATP. It can reduce the expression of P2X_7_ receptor, inhibit the conduction pathway of cell death, reduce the release of inflammatory factor IL-1*β*, and improve cell survival.

## 1. Introduction

Adenosine triphosphate (ATP) is the main life energy source; it supports the physiological activities of organisms including human beings [1–3]. Studies in the past few years have shown that sustained high extracellular concentrations of ATP can damage surrounding cells and becoming dangerous signaling molecules. Therefore, the role of ATP-P2X purine signaling pathway in cerebral ischemia-reperfusion injury has attracted much attention.

Pyroptosis is a form of cell death. Recent studies have shown that when caspase-4/5 (humans) recognizes pathogen mode molecules or human danger signal molecules, cells, caspase-1, and caspase-11 (mice) could activate and cleave Gasdermin D protein, resulting in the formation of cell membrane pores, the release of inflammatory factors, and finally cell lysis and death. In recent years, many cellular and animal experiments have shown that progesterone could reduce edema after cerebral ischemia and inhibit inflammatory cascade.

48 hours after cerebral ischemia in rats, progesterone could effectively inhibit the downregulation of tight junction protein expression, maintain the integrity of the blood-brain barrier, and reduce brain edema [4]. Cai et al. [5] found in the rat model of experimental subarachnoid hemorrhage that progesterone can reduce acute brain injury by reducing apoptosis and inhibiting oxidative stress.

Progesterone treatment can improve the neurological function of rats with brain injury, and its mechanism may be related to the regulatory of progesterone on immune-inflammatory after brain injury [6]. In animal experiments of acute toxic injury, traumatic injury, spinal cord injury, and the central nervous system stroke, the application of progesterone therapy can delay the necrosis and apoptosis of nerve cells in model animals, reduce the inflammatory reaction and brain edema caused by ischemic brain injury, promote the synthesis of brain myelin sheath, and promote the reconstruction of the blood-brain barrier [7–9].

How to select the right cells and observe the regulation of progesterone in the state of scorch death of neurons?

SH-SY5Y cells are derived from the neural crest during neural development and exhibit biochemical, pharmacological, and functional properties similar to those of neurons. It provides a good in vitro model for studying neuronal function, differentiation, and death.

In the paper, SH-SY5Y cells were used to observe ATP-induced cell and the mechanism of progesterone.

## 2. Related Works

### 2.1. Cell Line

Human neuroblastoma SH-SY5Y cell line was supported by the typical cell substrate library of Shanghai Academy of Sciences, Shanghai.

### 2.2. Reagents

DMEM culture substrate was purchased from HyClone. Fetal bovine serum was purchased from Sijiqing Co. Cell Counting Kit-8 (CCK-8), RPIA lysate, and ECL luminescence reagent were purchased from Biyun Tian Co. Streptomycin and penicillin mixture (100×), fetal bovine serum (FBS), and phenylmethanesulfonyl fluoride (PMSF) were produced by Solarbio Co., and GAPDH Rabbit Polyclonal Antibody was purchased from Xianzhi Co. P2RX7 antibody and caspase-1/P20/P10 antibody were purchased from Sanying Co. Caspase-11 (17D9) Rat mAb was purchased from Cell Signaling Technology (CST). 10∗SDS PAGE Running Buffer was purchased from Bomaide Co. Prestaining Protein Marker was purchased from Thermo Fisher Scientific.

### 2.3. Cell Culture

Human neuroblastoma cell line SH-SY5Y was cultivated in a 5% CO_2_ saturated humidity incubator at 37°C with Dulbecco's modified Eagle's medium (DMEM). SM (100 U/mL), PNC (100 U/mL), and 10% FBS were added to the medium. Change DMEM every 48 h intervals. SH-SY5Y cells were subcultured after monolayer cells fusion and then randomly divided into control group, BBG group, ATP group, and progesterone+ATP group.

### 2.4. Cell Viability Check

#### 2.4.1. Grouping

SH-SY5Y cells were routinely cultured in the blank without medicine. In the ATP part, cells were cultured with different concentrations of 1, 3, 6, or 9 mmol/L ATP for 2 h. The cells in the progesterone+ATP group were incubated in the medium containing 3, 10, 30, and 100 nmol/L progesterone for 30 min and then incubated in the medium containing ATP (concentration of 6 mmol/L) for 2 h.

#### 2.4.2. Measure

Logarithmic-phase human neuroblastoma SH-SY5Y cells (3 × 10^4^) were incubated in consistent temperature of 37°C and 5% CO_2_ for 24 hours. The saturated humidity incubator was placed in a 96-well plates in 100 *μ*L culture medium. Then, the medium with ATP at the indicated concentration (1, 3, 6, or 9 mmol/L) was replaced with the previous medium. After ATP incubated the cells for 2 h, the cells were incubated in dark, and 10 cells were added to each well 10 *μ*L CCK-8 solution for 2 h. The absorbance (A) at 460 nm was detected by ELISA. The cell viability was calculated by the average of three A values. The calculation formula is cell viability (%) = [A (dosing) − A (blank)]/[A (not dosing) − A (blank)] × 100%. Each group had 3 parallel wells, and the experiment was repeated 3 times.

#### 2.4.3. Western Blot

The expression of the cell pyroptosis-related protein was detected by Western blot assay. Grouping is as follows: in the control group, SH-SY5Y cells were cultured without any drugs. In the DMSO group, the final concentration of DMSO was 0.01% by adding DMSO to the culture medium, which was consistent with the final concentration of dissolve progesterone, so as to eliminate the possibility of the influence of related protein. In the BBG group, the effective concentration of brilliant blue G (BBG) in the medium reached 1 mmol/L, which inhibited the expression of P2X_7_ receptor's expression. In the ATP group, the cells were incubated in different concentrations (1, 3, 6, and 9 mmol/L) of ATP for 2 h. In the progesterone+ATP group, the cells were preincubated with different concentrations (3, 10, 30, and 100 nmol/L) of progesterone for 30 min and then incubated in ATP (concentration of 6 mmol/L) medium for 2 h. The expression of purinergic P2X_7_ receptor, caspase-1, caspase-11, and IL-1*β* was assessed.

## 3. Results

### 3.1. Survival of SH-SY5Y Cells Induced by Different Concentrations of ATP for 2h

SH-SY5Y cells were inoculated into 96-well plates and treated with different treatment factors according to the experimental grouping requirements. When the cells are in logarithmic growth phase, using the cell proliferation toxicity assay, 10 *μ*L of CCK- solution was added to each well at 37°C and incubated in the dark for 2 h, and the absorbance of each well was detected at the wavelength of 450 nm with enzyme labeling instrument. The calculation formula is as follows: cell viability (%) = [A (dosing) − A (blank)]/[A (not dosing) − A (blank)] × 100%. In this experiment, the cell survival rate of the control group was 100%.

First, we choose different concentrations of ATP to act on the cell. The drug concentrations of ATP are 1, 2, 3, 4, 5, 6, 7, 8, and 9 mmol/L or 10 mmol/L, respectively. We found that with the increase of drug concentration, the cell survival rate decreased gradually, with obvious drug dependence. When 6 mmol/L ATP was used on the cell, the survival rate of the cell was reduced to 55.4%, reaching the half lethal dose of the cell. Through this method, the best dose to make SH-SY5Y cells reach the median lethal dose was selected (Table 1).

In this experiment, a series of concentration gradients of ATP were set, including 1 mmol/L, 3 mmol/L, 6 mmol/L, and 9 mmol/L. The results showed that the survival rates of SH-SY5Y cells treated with different concentrations of ATP for 2 h were 97.98%, 84.53%, 55.4%, and 34.99%, respectively, and 100% in the normal control group. However, with the increase of ATP concentration, the cell survival rate decreased gradually in a dose-dependent manner. There were significant differences in cell survival rate between the two groups (*P* < 0.01). The cell survival rate of ATP at the concentration of 6 mmol/L was 55.4% when the concentration of ATP was 6 mmol/L. This result is consistent with that of the preexperiment. The results showed that the median lethal dose of ATP was 6 mmol/L (Figure 1).

### 3.2. Effect of Progesterone on the Survival Rate of ATP-Induced SH-SY5Y Cells

Different concentrations of progesterone (3, 10, 30, or 100 nmol/L) SH-SY5Y cells were preincubated with different concentrations of progesterone (3, 10, 30, or 100 nmol/L) for 30 min, and then the substrate containing 6 mmol/L ATP was used to replace the cell culture substrate for 2 h. The results of CCK-8 showed that the cell energy of ATP group was 55.4% and reached the median lethal dose when the cell survival rate of control group was 100%. In the progesterone+ATP groups, the progesterone (3, 10, 30, or 100 nmol/L) +ATP (6 mmol/L) groups were 50.22%, 55.46%, 70.54%, and 55.97%, respectively. When the concentration of progesterone was in the range of 30 nmol/L, the cell viability increased with the increase of concentration of progesterone. The cell viability reached the peak when the concentration of progesterone was 30 nmol/L. With the further increasing of progesterone concentration to 100 nmol/L, the cell viability decreased significantly. The protective effect of progesterone on cells was the strongest at 30 nmol/L (Figure 2).

### 3.3. The Expression of Associated Proteins of Pyroptosis Were Evaluated by Western Blot Assay

The expression of purinergic P2X_7_ receptor, caspase-1, caspase-11, and IL-1*β* were assessed by western blot assay (Figure 3(a)). There were no significant changes in the expression of IL-1*β*, caspase-1, and P2X_7_ receptor in the control group, DMSO group, and BBG group. Their expressions of ATP in SH-SY5Y cells increased significantly after ATP conduction for 2 h (*P* < 0.01). There was no significant change in caspase-11 (*P* > 0.05) (Figure 3(d)), an important protein of the nonclassical pastway of pyroptosis.

In the progesterone+ATP group, the expressions of IL-1*β*, caspase-1, and P2X_7_ acceptor were significantly lower than that of ATP (*P* < 0.01). Therefore, progesterone can inhibit ATP-induced cell pyroptosis (Figures 3(b), 3(c), and 3(e)). The expression of P2X_7_ receptor in the control group, DMSO group, and BBG group had no significant changes in the nonclassical pathway-related proteins caspase-11 and IL-1*β*. As a comparison to the blank part, P2X_7_ showed that the expression of the receptor protein was upregulated after 2 hours of ATP action. There was no significant difference in the expression of caspase-11, the key protein of noncanonical pathway (*P* > 0.05).

The expression of P2X_7_ receptor protein was downregulated after progesterone preculture for 30 min and ATP treatment for 2 h. There was no significant change in the expression of caspase-11, showing no statistical significance (*P* > 0.05).

## 4. Experimental Analysis

The regulation and mechanism of cell pyroptosis are different from cell death ways such as necrosis and apoptosis, which provides a new idea for clinical prevention and treatment.

### 4.1. Cell Pyroptosis

The pyroptosis pathway refers to the programmed cell death based on activation of inflammasome. The pore size of the membrane formed by pyroptosis is between 1 and 2 nm. Thus, the cell membrane loses its integrity and cannot regulate the entry and exit of substances. Finally, the cell membrane dissolves and releases the cell contents and further induces the inflammatory reaction of other cells [10, 11]. There are two types of cell pyroptosis, caspase-4/-5/-11-dependent nonclassical access and caspase-1-dependent canonical access [12, 13] (Figure 4).

#### 4.1.1. Typical Cell Apoptosis pathway

In the typical apoptosis pathway, apoptosis-related speck-like protein including a CARD can indirectly connect pattern recognition acceptors (NLRP1, NLRP3, AIM2, Pyrin, etc.) with cysteine protease-1 (pro-caspase-1), cysteine protease-1 to form a polymeric complex, namely, inflammasome or caspase-1-dependent inflammasome. Researchers also found that NLRP1 and NLRC4 could directly connect to caspase-1 independent of ASC [14]. When inflammasomes such as NLRP3, NLRC4, Aim2, and Pyrin are activated, they will form active caspase-1 by activating and cleaving pro-caspase-1. Caspase-1 can form active N-terminal and C-terminal by cleaving gasdermin D. And the N-terminal can promote cell death and cell membrane perforation. At the same time, activated IL-1*β* is formed through the split of pro-IL-1*β* by caspase-1 and released extracellular, expanding the inflammatory response [12, 15].

#### 4.1.2. Nonclassical Pyroptosis Access

In the nonclassical pyroptosis access, LPS could directly adhere to caspase-4/-5/-11 straight away. On the one hand, activated caspase-4/-5/-11 can lyse gasdermin D protein, and the N-terminal of gasdermin D could mediate cell membrane lysis and pyroptosis and also excite NLRP3 inflammasomes to activate caspase-1 and then produce IL-1*β* and release. On the other hand, activated caspase-4/-5/-11 activates pannexin-1 and releases ATP to open the membrane channel P2X_7_, resulting in cell membrane pores formation and inducing cell pyroptosis. Activated pannexin-1 also activates NLRP3 inflammasomes by releasing K^+^, which eventually produces IL-1*β* and releases it externally [16].

### 4.2. Possible Mechanisms of Cell Pyroptosis Induced by Extracellular Persistent High Concentration of ATP

Studies have shown that P2X_7_R plays an important role in the occurrence and development of a variety of central nervous system diseases. After traumatic or ischemic brain injury, ATP and degradation products released from local damaged cell would spread to adjacent areas. It will continuously stimulate glial cells in the damaged and adjacent areas, lead to glial cell activation, and increase the expression of P2X_7_R [17].

In recent years, most studies were to explore the neuroprotective effect of progesterone on brain injury and its possible mechanism in animal models and rarely explore the effect of progesterone on nerve cells. Therefore, the focus of this experiment is to take neuroblastoma cell SH-SY5Y as the research object to explore whether the effect of progesterone on ATP-induced SH-SY5Y cell injury is related to the change of P2X_7_R. There are many reports on the expression of P2X_7_R in glial cells, and the existence of P2X_7_R in SH-SY5Y cells has been confirmed in the literature [18].

Some studies showed that the degree of peripheral nerve injury with P2X knockout mice was significantly less than the normal mice, and the pain sensitivity decreased as well. It is a common phenomenon that the activation of P2X_7_R by elevated ATP concentration in a variety of secondary injury of central or peripheral neurons, and the protective effect of progesterone on secondary injury of neurons has also been confirmed. It is not a coincidence that progesterone and ATP are significantly increased at the site of brain injury. This experiment conducted a detailed study to expose whether progesterone can slow down the focal death of SH-SY5Y cells induced by high concentration ATP by regulating the activation of P2X_7_R.

Pyroptosis mainly occurs in macrophages, but it also occurs in microglia [19]. Purinergic P2X_7_ receptors are activated in response to high release of ATP under pathological conditions (such as hypoxia or cell disintegration). They are associated with the inflammatory and injurious responses of organisms to these pathological incidents [20, 21].

Caspase-1 activates and cleavages gasdermin D protein when extracellular persistent high concentration of ATP acts on P2X_7_ receptors in SH-SY5Y cells. The active N-terminal of Gasdermin D protein can perforate the cell membrane and form cell membrane pores, allowing the passage of various cations and organic substances below 900 D. High concentration of ATP activates P2X_7_ receptor and induces a large amount of Ca^+^ influx, K^+^ outflow, and the discharge of proinflammatory cytokine IL-1*β*. Cell pyroptosis occurs as a result. Inhibition of P2X_7_ receptor activation can reduce cell excitability and thereby reduce cell death.

### 4.3. Protective Effect of Progesterone on ATP-Induced Pyroptosis of SH-SY5Y Cells

#### 4.3.1. Possible Mechanisms of Neuroprotective Effect of Progesterone

The level of progesterone in blood increases rapidly following brain injury, which suggests progesterone is related to the repair of damaged nerve [20]. Animal experiments have shown that brain edema mainly occurs 3 hours after ischemia reperfusion. The expression of aquaporin-4 (AOP-4) around the lesion was decreased after intraperitoneal injection of progesterone, and vasogenic brain edema at the lesion site was reduced as well. It is generally believed that the nongenetic effect on cell membrane receptors contributes to the neuroprotective effect of progesterone. It changes the biological activity of neurons and regulated the neurotransmitter receptors and ion channels. Progesterone can regulate the nervous system's function and structure through neurotransmitter receptors on neurons and glial membranes [22]. After brain injury, a large number of cytokines (IL-1*β*) released would cause inflammation, and progesterone can inhibit the release of these cytokines, hence reducing brain edema.

Many animal model experiments show that progesterone can improve age-related neurodegenerative diseases such as Alzheimer's disease [23] and Parkinson's disease [24]. In the animal experiment of brain injury in rats, progesterone can reduce caspase-3 activity and apoptosis [25]. Lockhart et al. [26] found that pretreatment with low concentration of progesterone metabolite allopregnanolone could reduce the number of apoptotic cells in a dose-dependent manner in the in vitro apoptosis model induced by N-methyl-D-aspartic acid. Hoffman et al. [27] also found that low-dose progesterone can significantly reduce seizures in ovariectomized rats. The mechanism is still unknown, although a large number of animal experiments have confirmed the neuroprotective effect of progesterone.

Brain ATP is mainly released by glial cells having neurotransmitter activity, so it is called glial neurotransmitter. Under physiological conditions, the concentration of intracellular ATP reaches mmol/L and extracellular ATP *μ*mol/L level. Extracellular ATP at mmol/L level would activate P2X_7_R, form cation channel, mediate Ca^2+^, Na^+^ influx, and K^+^ outflow, depolarize cells, and maintain normal excitatory activity of nerve cells. Under the pathological conditions of brain injury, cerebral ischemia, and inflammation, the glial cells in the injured area release a large amount of ATP and its degradation products, spreading to the adjacent areas. High concentration ATP stimulates P2X_7_R on the cell membrane consistently, forming a “membrane pore” that allows various cations and organic substances below 900 d to pass through, resulting in the imbalance of the homeostasis of the intracellular environment and death. The formation of membrane pores can accelerate Ca^2+^ influx, cause calcium overload, release inflammatory factors from glial cells, then trigger inflammatory reaction, and aggravate brain tissue damage [28]. Suadicani et al. [29] used the human glioma 1321N1 cell line expressing P2X_7_ receptor as the experimental object and found that benzoyl benzoate adenine nucleoside triphosphate can significantly increase the intracellular Ca^2+^ concentration, YO-PRO-1 uptake, and ATP release. Studies have shown that ATP acts on differentiated NG108-15 nerve cells. It not only causes intracellular calcium overload but also mediates calcium release through inositol triphosphate receptor after activating P2X_7_ receptor, resulting in cell apoptosis [30]. Therefore, calcium overload is also an important factor for the toxic effect of P2X_7_R. The protective effect of progesterone on secondary injury of neurons has been confirmed by common activation of P2X_7_R through elevated ATP concentration. There are no reports yet to study whether progesterone can intervene by regulating the activation of P2X_7_R and what is the neuroprotective effect of ATP-induced secondary brain injury.

#### 4.3.2. Progesterone Has a Protective Effect on ATP-Induced Pyroptosis of SH-SY5Y Cells

In this study, neuroblastoma SH-SY5Y cells were used to observe the effect of progesterone on ATP-induced SH-SY5Y cell injury and to explore the role of P2X_7_R in progesterone neuroprotection. The results of CCK-8 showed that the cell survival rate decreased with the increase of ATP concentration in a dose-dependent manner. SH-SY5Y cells were pretreated with four different concentrations of progesterone before ATP. The results of cell survival showed that compared with the experimental group supplemented with ATP, the cells were pretreated with 3, 10, 30, and 100 nmol/L progesterone, respectively, and then, the same dose of ATP was added to the experimental group.

The results of CCK-8 experiment showed that the cell survival rate decreased with the increase of ATP concentration in a dose-dependent manner (Figure 1 and Table 1). The results showed that there was no significant difference in cell survival rate between 3 nm progesterone+ATP group and ATP group (*P* > 0.05), but the protective effect was the most significant when the concentration of progesterone increased to 30 nm. When the concentration of progesterone continued to increase, the cytoprotective effect was not further enhanced but decreased compared with the 30 nm progesterone+ATP group (Figure 2). It shows that progesterone can protect the focal death of brain nerve cells induced by ATP in a certain concentration range.

We further detected the expression of P2X_7_R protein by Western blotting (Figures 3(a) and 3(b)). Another P2X_7_R-specific blocker BBG was used in the experiment. There was no significant difference identified between BBG pretreatment and normal control group, indicating that the activation of P2X_7_ receptor plays a key role in the change of membrane permeability of SH-SY5Y cells induced by ATP, while progesterone has the effect of P2X_7_ receptor blocker and inhibits the increase of membrane permeability induced by ATP. It was found that the protein expression in ATP group was significantly higher than that in the normal control group (*P* < 0.01); and protein in progesterone+ATP group was significantly lower than that in ATP group (*P* < 0.01).

The progesterone could inhibit ATP-induced P2X_7_ receptor expression, to reduce the discharge of inflammatory element IL-1*β*, prevent cell pyroptosis, and reduce cell mortality. Western blot results showed that extracellular high concentration of ATP could not activate caspase-11, a noncanonical pyroptosis pathway-related protein in SH-SY5Y cells. Progesterone can inhibit the expression of P2X_7_ protein induced by ATP in SH-SY5Y cells, protect against the formation of cell membrane pore, and inhibit the formation of cell pyroptosis. It can also reduce cell apoptosis and cell mortality through impediment release of IL-1*β* inflammatory cytokines (Figures 3(d) and 3(e) and 4).

This study suggests that progesterone protects SH-SY5Y cells from injury induced by high concentration of extracellular ATP. Progesterone can inhibit the activation of P2X_7_R, prevent the formation of membrane pores, and reduce the permeability of cell membrane, hence to reduce cell focal death rate. It provides a theoretical basis for progesterone in brain protective therapy as a potential molecular mechanism to protect injured neurons.

## 5. Conclusion

### 5.1. Cell Scorch Death May Be Beneficial to Inhibit Infection

Several studies have shown that the expression of caspase-1/-11 and its mediated release of inflammatory factors and cell death help to inhibit infection (including acute enteritis in mice induced by dextran sodium sulfate DSS) and accelerate tissue repair [31]. Cell scorch death is conducive to the release of intracellular pathogens, which can be swallowed, killed, and cleared by other phagocytes, in order to prevent the reproduction and persistence of pathogens in cells [32]. Therefore, it can activate the inflammatory bodies and scorch death the infected cells (or activated cells), strengthen the local inflammatory response, accelerate the clearance of heat sources (pathogenic microorganisms and innate immune cells activated by PAMP), and promote the repair of damaged tissues and the recovery of diseases.

### 5.2. Cell Scorch Death May Be Beneficial to Reduce Chronic Inflammatory Diseases

Pyrosis is one of the important exit mechanisms for activated macrophages. When macrophages continue to activate without focal death, their immune metabolic pathways would be changed, resulting in lipid deposition and foam cells or fat macrophages. And the cells would consistently secrete inflammatory factors and chemokines, leading to more immune cells to focus tissue, which increases the risk of chronic inflammatory diseases such as atherosclerosis and obesity [33].

The formation of membrane pores induced by extracellular ATP is regulated by P2X_7_ receptor. Studies have found that when bacterial infection or tissue damage occurs, host cells and bacterial cells can release ATP from intracellular to extracellular [34]. The extracellular ATP can be used as the second signal of NLRP3 inflammatory body activation; it can induce cell scorch death of innate immune cells, such as macrophages.

Pyrosis is regarded as an important result of ATP-induced activation of macrophage inflammatory bodies. It is an inflammatory cell death, which is manifested in the formation of some cell membrane channels or cell membrane pores, resulting in the release of intracellular inflammatory substances and cell rupture [35]. The interaction of extracellular ATP with receptors on the cell membrane, especially P2X_7_R, activates the inflammatory bodies induced by ATP [36]. When ATP binds to P2X_7_R, a nonselective cation channel will be formed, resulting in the release of K^+^. If P2X_7_R is continuously activated, pannexin-1 will be recruited to form membrane pores, resulting in IL-1*β* release and cell death. And ATP-induced K^+^ efflux will trigger the assembly of inflammatory body NLRP3, resulting in the activation of caspase-1. Activated caspase-1 cleaved gasdermin d to produce its N-terminal fragment. The fragment has membrane binding function and forms pores on the cell membrane. The inner diameter of the resulting membrane pores is about 32 nm [37], allowing mature IL-1*β*, HMGB1, and other intracellular components pass through [38], resulting in cell scorch death. Previous studies have found that ATP-P2X_7_R signal can integrate PI3K/Akt and AMPK mTOR signaling pathways, resulting in the death of tumor cells [39]. It confirms our speculation that the formation of ion channels and membrane pores induced by extracellular ATP is regulated by AMPK as well. Indeed, we found that the activity of mTORC1 was completely inhibited and AMPK was significantly activated during ATP-induced cell death.

In this experiment, the expression of P2X_7_R in SH-SY5Y cells is high, and P2X_7_R is used to study the involvement of receptors, signal pathways, and key signal molecules in ATP-induced focal death of SH-SY5Y cells and to examine the molecular action mechanism of progesterone, so as to reliably clarify the role of progesterone and more evidence of the downstream signal pathway of P2X purine receptor. The specific molecular mechanism of progesterone inhibiting ATP-induced focal death of SH-SY5Y cells was verified.

The time effect and dose effect of ATP intervention on SH-SY5Y cells were observed. The expression of P2X_7_ was measured to detect the receptor protein in SH-SY5Y cells and the changes of P2X_7_. The receptor protein expression in SH-SY5Y cells induced by ATP was observed at different timestamps and concentrations.

The regulatory effect of ATP on P2X_7_ expression was verified by the receptor protein in SH-SY5Y cells. The regulation effect of progesterone on ATP-induced focal death of SH-SY5Y cells was further verified. It is confirmed that progesterone can inhibit ATP-induced pyroptosis of SH-SY5Y cells by regulating typical pyroptosis pathway-related proteins. The mechanisms could be that progesterone inhibits cell pyroptosis by inhibiting the expression of P2X_7_ protein, reduces cell permeability, and relates the expressions of related inflammatory cytokines IL-1*β* and caspase-1.

It is suggested that progesterone has a protective effect on SH-SY5Y cells induced by extracellular high concentration ATP. The mechanism is to reduce cell death by inhibiting P2X_7_R activation and reducing cell membrane permeability. The results offer an experimental basis for progesterone in the treatment of brain injury. It also provides a theoretical basis for screening neurosteroid-related drugs in the clinic.

## Figures and Tables

**Figure 1:** Effects of different concentrations of ATP for 2 h on the survival rate of SH-SY5Y cells. Mean ± SEM. *n* = 3. ^∗^*P* ≤ 0.05 and ^∗∗^*P* ≤ 0.01 vs. control group.

**Figure 2:** How dose progesterone regulate ATP-induced pyroptosis in SH-SY5Ycells. Mean ± SEM. *n* = 3. ^∗^*P* ≤ 0.05 and ^∗∗^*P* ≤ 0.01 vs. control group.

**Figure 3:** (a) Western blot assay used to detect protein levels, such as purinergic P2X_7_ receptor, caspase-1, caspase-11, and IL-1, and GAPDH was used as compared protein. (b) Effects of 30 nmol/L progesterone on the expression of P2X_7_ receptor in SH-SY5Y cells induced by 6 mmol/L ATP. Mean ± SEM. *n* = 3. ^∗^*P* ≤ 0.05 and ^∗∗^*P* ≤ 0.01 vs. control group. (c) Effect of 30 nmol/L progesterone on caspase-1 in SH-SY5Y cells induced by 6 mmol/L ATP. Mean ± SEM. *n* = 3. ^∗^*P* ≤ 0.05 and ^∗∗^*P* ≤ 0.01 vs. control group. (d) Effect of 30 nmol/L progesterone on caspase-11 in SH-SY5Y cells induced by 6 mmol/L ATP. Mean ± SEM. *n* = 3. ^∗^*P* ≤ 0.05 and ^∗∗^*P* ≤ 0.01 vs. control group. (e) Effect of 30 nmol/L progesterone on IL-1*β* in SH-SY5Y cells induced by 6 mmol/L ATP. Mean ± SEM. *n* = 3.^∗^*P* ≤ 0.05 and ^∗∗^*P* ≤ 0.01 vs. control group.

**Figure 4:** Diagram of the pyroptosis signaling pathway. (a) Nonclassical pyroptosis access and (b) canonical pyroptosis access.

**Table 1:** Effects of different concentrations of ATP on the cell survival of the SY5Y cells.

ATP	Cell survival (%)	*P*
Control	100	—
1	97.98 ± 0.044^∗∗^	0.008
2	92.10 ± 0.92^∗∗^	0.022
3	84.53 ± 4.81^∗∗^	0.001
4	77.63 ± 0.67^∗∗^	0.016
5	68.93 ± 0.55^∗∗^	0.006
6	55.40 ± 3.79^∗∗^	0.016
7	49.33 ± 0.55^∗∗^	0.002
8	42.47 ± 0.71^∗∗^	0.003
9	34.99 ± 4.46^∗∗^	0.008
10	21.40 ± 0.82^∗∗^	0.002

Values were presented as mean ± SD. ^∗^*P* < 0.05 and ^∗∗^*P* < 0.01, compared to the control group.

## Data Availability

No data were used to support this study.
